The article "Applicability of Moorrees, Fanning, and Hunt Method for Age Estimation in Gandhinagar, India: An Orthopantomogram (OPG)-Based Retrospective Study" was retracted in 2025. Reasons: no approval from a third party; copyright claims; concerns about the results or conclusions.

# Applicability of Moorrees, Fanning, and Hunt Method for Age Estimation in Gandhinagar, India: An Orthopantomogram (OPG)-Based Retrospective Study

**DOI:** 10.7759/cureus.83743

**Published:** 2025-05-08

**Authors:** Megha C Patel, Foram Patel, Shubham S Srivastav, Disha Makwani, Chhaya Patel, Miral Mehta, Chandni J Adalja, Khushi Rathod

**Affiliations:** 1 Department of Pediatric and Preventive Dentistry, Karnavati School of Dentistry, Karnavati University, Gandhinagar, IND; 2 Department of Periodontology, Ganga Dental Clinic, Vadodara, IND; 3 Dentistry, Government Dental College and Hospital, Ahmedabad, IND

**Keywords:** age determination, chronological age, dental age, forensic odontology, tooth developmental stages

## Abstract

Background: Age estimation is crucial for human identification in forensic investigations and humanitarian efforts. Tooth development provides one of the most accurate ways to determine age, showing remarkable consistency regardless of external conditions. The Moorrees, Fanning, and Hunt (MFH) technique assesses dental growth by examining the formation of crowns, roots, and apex completion. This method has proven reliable through numerous studies spanning different ethnic and geographic groups. Its systematic approach and scientific foundation make it an invaluable tool in modern forensic odontology, enhancing the accuracy of age estimation practices.

Aim: The study aims to evaluate the applicability of the MFH methods to estimate dental age and to compare it with the chronological age of the children in the population of Gandhinagar in the state of Gujarat, India.

Materials and methodology: A retrospective study was carried out to assess the dental age of the patients visiting the Karnavati School of Dentistry, Gandhinagar, for dental check-ups. Panoramic radiographs were obtained from the archives of the database that have been taken from January 2020 till August 2023 for study purposes and were examined to fit into inclusion criteria. The sample included 388 orthopantomograms (OPGs) of children aged two to 12 years. Each child’s tooth was assessed based on developmental stages outlined in the MFH method. Statistical analysis was done using IBM SPSS Statistics for Windows, Version 27 (IBM Corp., Armonk, NY). Simple linear regression was used to formulate a regression model to determine the correlation between chronological age and dental age.

Results: The MFH method consistently underestimated dental age (DA) compared to chronological age (CA) across both genders. Analysis of 388 subjects showed male individuals (n = 233) had a mean DA of 6.822 years versus CA of 7.559 years (underestimation: 0.74 years, p<0.001), while female individuals (n = 155) had a mean DA of 6.337 years versus CA of 7.049 years (underestimation: 0.71 years, p = 0.011). Both genders showed strong positive correlations (male individuals: ρ = 0.974, female individuals: ρ = 0.980) and linear relationships (male slope (b) = 1.026, female slope (b) = 1.029) with chronological age, where female participants demonstrated slightly earlier dental maturation patterns.

Conclusion: The MFH method consistently underestimates dental age when compared to chronological age, indicating that it may lack accuracy in dental age assessment in the Gandhinagar population.

## Introduction

Age estimation holds a pivotal role in forensic science and stands as one of the most intricate aspects of human identification [1]. Forensic odontology is a specialized branch of forensic medicine that focuses on the accurate examination, documentation, and presentation of dental evidence to support legal proceedings and the pursuit of justice. [2]. Forensic odontology plays a crucial role in circumstances where habitual methods of identification, such as fingerprinting and visual recognition, cannot be performed in cases of decomposed, charred, or skeletonized bodies [3].

The estimation of chronological age through dental examination has gained substantial importance in contemporary forensic practice. This methodology finds extensive application across numerous forensic scenarios, including criminal investigations where age determination is crucial for legal proceedings, mass disaster victim identification requiring rapid and accurate age assessment, evaluation of age claims in asylum seekers, resolution of civil disputes involving age-related matters, archaeological studies necessitating age determination of historical remains, and various legal proceedings where age verification is essential for justice administration [4].

Dental age estimation encompasses three life phases: prenatal/neonatal, children/adolescent, and adult. Major methods for children include Schour and Masseler's developmental charts (1941), Nolla's 10-stage evaluation (1960), Demirjian's sex-specific scoring system, Cameriere's open apex measurements, and Moorrees, Fanning, and Hunt's (MFHs) 14 mineralization stages (1963), each offering distinct approaches to age assessment [5,6].

The MFH method, established in 1963, represents a groundbreaking and comprehensive approach to dental age estimation. This methodology introduces a systematic analysis of tooth mineralization stages, encompassing the entire developmental sequence from initial cusp formation through complete root apex closure. The method provides a detailed framework for age assessment based on dental development patterns, offering a scientific foundation for forensic age estimation practices [7,8].

Orthopantomograms (OPGs) enable comprehensive dental age assessment by capturing the entire dental arch in a single image, surpassing intraoral radiographs. By examining tooth eruption patterns, root development stages, and resorption, dentists can estimate age using established development charts. This non-invasive and painless radiographic technique is widely accessible, making it a preferred choice for dental age estimation. The method is especially reliable for assessing younger individuals' ages due to their rapid and predictable dental development, though accuracy may decrease in older adults [9,10].

Recent technological advancements, particularly in digital imaging and statistical analysis, have enhanced the precision of forensic age estimation. The integration of digital pantographs and software enhancements, such as Adobe Photoshop (Adobe, San Jose, CA) for a detailed comparison of developmental stages, combined with population-specific standards, has significantly improved measurement accuracy while maintaining fundamental methodological principles. These innovations have strengthened the reliability of age estimation in modern forensic odontology [11,12].

Dental age estimation using the MFH method has emerged as a critical forensic tool, blending advanced technological capabilities with precise scientific methodology. Practitioners require deep expertise in dental development patterns, radiographic interpretation, and statistical analysis to effectively apply this technique [13,14].

## Materials and methods

Rationale

Reliable age estimation plays a vital role in forensic science, legal matters, and clinical dentistry. While the MFH method is a well-established approach for dental age estimation, its accuracy may differ across populations due to genetic and environmental influences. Therefore, it is essential to evaluate its effectiveness within the Gandhinagar population. This study seeks to examine the relationship between dental age and chronological age, ensuring more precise forensic age estimation and enhancing its application in clinical and legal contexts.

Null hypothesis

The null hypothesis tested was: "We hypothesize that there will be no significant difference between dental age and chronological age of children in the Gandhinagar population."

Study design and ethical approval

A radiographic-based retrospective study was carried out in the Department of Pediatric and Preventive Dentistry, Karnavati School of Dentistry, Karnavati University, Gandhinagar.

Archived radiographic data were used with official approval, ensuring confidentiality, anonymity, and compliance with ethical research standards. all data included in the study was retrospective and collected from the relevant children with full consent of the parents/guardians, who were informed that the medical data could be used for scientific study under strict conditions of anonymity. all radiographic analysis of children was conducted as it was required for diagnostic or treatment planning purposes.

Sample collection

Assuming the division in the proportion of genders in the specified age group to be 50%, as commonly observed in the population, at a 5% confidence interval, the sample size was calculated to be 384. Considering a minimum 5% rate of attrition due to ineligibility, a total of 420 subjects were included in the study.

A total of 420 OPGs (247 male and 173 female subjects) of healthy children (aged from 2.00 to 14 years) were obtained with official approval from the Department of Oral Medicine and Radiology, Karnavati School of Dentistry database from January 2020 to August 2023. Of these, 32 were excluded based on predefined exclusion criteria, resulting in a final sample size of 388. These 388 OPGs were subsequently analyzed for the interpretation of results and were examined to fit into inclusion criteria.

Inclusion criteria

OPGs of children aged two to 14 years, including all complementary sets of teeth appropriate for that age group, were selected for inclusion. Only diagnosable OPGs with clear images, free from faults or blurriness, were considered.

Exclusion criteria

OPGs of children and subadults below two years and above 14 years were excluded from the study. Additionally, any cases with developmental anomalies or pathologies were not considered. OPGs of children lacking initial details such as date of birth, gender, and address were also excluded.

Parameters evaluated

Chronological age estimation: The patient's chronological age was determined by calculating the time interval between their birth date and the date when their OPG was taken, expressed in years.

Dental age estimation: To assess dental age, researchers evaluated each existing lower jaw tooth individually using the MFH chart guidelines [7]. They then computed the average age based on all present mandibular teeth. This calculated dental age was subsequently evaluated against the previously determined chronological age.

Assessment of dental age using the MFH method

The dental age estimation was performed by direct comparison of tooth developmental stages observed on panoramic radiographs with the standards established by the MFH method.

The developmental phases of tooth formation are illustrated in separate figures, each highlighting specific aspects of dental growth. Figure 1 depicts the formation stages of teeth with a single root, while Figure 2 illustrates the developmental progression of teeth with multiple roots.

Table 1 presents the stages of tooth formation along with their corresponding coded symbols.

Additionally, the developmental norms for permanent upper and lower incisor teeth are shown in distinct diagrams, with Figure 3 representing male subjects and Figure 4 displaying the corresponding developmental patterns for female subjects.

The norms for the development of posterior teeth in male subjects and the permanent maxillary and mandibular canines in female subjects are depicted in Figure 5 and Figure 6, respectively.

A total of seven mandibular teeth (I-M2) were examined, and their developmental status was determined based on charts provided by Moorrees, Fanning, and Hunt. The developmental stages of each tooth, from C-M2, were recorded and computed in years. These charts allowed for the direct representation of individual children's tooth formation using standard scores. Researchers assessed the developmental ratings of each tooth using OPGs, enabling comparisons of tooth maturation within the same child.

The charts were systematically divided into sections, each dedicated to a particular tooth. Horizontal bars represented the chronological development of each stage, incorporating distinct symbols to indicate the mean age of attainment, along with one and two standard deviation limits. Age scales were positioned at both the top and bottom of the charts for reference. The assessment of tooth formation was recorded by marking checkmarks for each tooth at its respective developmental stage. A vertical line drawn through corresponding points on the age scales facilitated the reading of tooth development ratings in standard scores at their intersections with horizontal bars.

To determine each patient’s dental age, the collected values were summed to generate an overall maturity score. For molar teeth, the mean age of the mesial and distal roots was computed separately and considered accordingly.

Statistical analysis

The data management and statistical analysis were conducted using Microsoft Excel 16 (Microsoft Corp., Redmond, WA) for data entry and IBM SPSS Statistics for Windows, Version 27 (IBM Corp., Armonk, NY) for analysis. The numerical data were represented as mean and proportions. The level of significance was kept to be 5%.

The normality was assessed with the Shapiro-Wilke test, which was significant, hence nonparametric tests were used. To assess the disparity between dental age (an estimated age) and chronological age (the true age) of the mandibular teeth, the study employed the Mann-Whitney U test. This analysis facilitated a comparison of the mandibular arches across all age categories as well as within distinct age groups for both genders. The findings were summarized using descriptive statistics and presented with a 95% confidence interval.

The connection between chronological age and dental age was assessed through the use of Spearman's correlation coefficient and univariate linear regression analysis. These statistical methods offered valuable insights into the relationship and predictive link between actual ages and their estimates.

## Results

According to the sample size distribution analysis (Table 2), the 388 participants (233 male and 155 female subjects) were distributed across age groups ranging from two to 14 years. The largest cohorts were observed in the six to seven and nine to 10-year groups, while the 12-14-year range had the fewest subjects. Male subjects predominated in most age categories, although a more balanced or female-skewed distribution was noted in some groups, such as five to six and seven to eight years. This age and gender spread provides a representative sample for evaluating developmental trends in the studied population.

**Table 1:** Sample-size distribution.

Age	Male	Female	Total
2-3	3	9	12
3-4	5	7	12
4-5	25	11	36
5-6	26	29	55
6-7	34	24	58
7-8	24	31	55
8-9	32	13	45
9-10	44	21	65
10-11	25	14	39
11-12	15	6	21
12-13	6	2	8
13-14	5	2	7
14	3	4	7
Total	233	155	388

Based on the descriptive analysis (Table 3), the MFH method produced an average dental age of 6.63 years, compared to a mean chronological age of 7.36 years. This difference was statistically significant (p = 0.002), indicating a tendency of the MFH method to underestimate age.

**Table 2:** Mean and standard deviation of dental and chronological age using the Mann-Whitney U test. * p-value is statistically significant and was calculated using the Shapiro-Wilk test for comparing dental and chronological age; (p-value <0.05).

Variable	N	Mean (years)	Standard deviation
Dental age	388	6.628	2.283
Chronological age	388	7.355	2.408
Paired t-test p-value			0.002*

Gender-based analysis (Table 4) indicated consistent underestimation of age using the MFH method in both sexes. Among male subjects (n = 233), the mean dental age was 6.82 years (SD = 2.11), compared to a mean chronological age of 7.56 years (SD = 2.24), with a statistically significant difference (p < 0.001). For female subjects (n = 155), the mean dental age was 6.34 years (SD = 2.50), while the chronological age averaged 7.05 years (SD = 2.62), also showing a significant difference (p = 0.003). Although males had higher average ages, female subjects exhibited greater variability, as reflected in their standard deviations.

**Table 3:** Mean values and variability of dental and chronological age analyzed with the Mann-Whitney U test for male and female subjects. * p-value is statistically significant for males and was calculated using the Shapiro-Wilk test comparing dental and chronological age between male and female subjects.

Gender	Variable	N	Mean (years)	Standard deviation
Male	Dental age	233	6.822	2.109
	Chronological age	233	7.559	2.243
	Paired t-test p-value			< 0.001
Female	Dental age	155	6.337	2.502
	Chronological age	155	7.049	2.615
	Paired t-test p-value			0.003*

In Table 5, the difference between dental age estimated using the Moorrees, Fanning, and Hunt (MFH) method and chronological age (CA) was assessed across genders. Male subjects showed an average underestimation of 0.737 years (SD = 2.17), which was statistically significant (p < 0.001). Similarly, female subjects exhibited an average underestimation of 0.712 years (SD = 2.55), also statistically significant (p = 0.011). These results indicate that the MFH method consistently underestimates age in both sexes.

**Table 4:** Mean difference, standard deviation, and p-value by using the Mann-Whitney test in male and female subjects. * p-value is statistically significant for males and was calculated using the Mann-Whitney test between male and female subjects. MFH: Moorrees, Fanning, and Hunt; CA: chronological age.

Gender		Paired difference		p-value
		Mean	Standard deviation	
Male	Age by MFH – CA	-0.737	2.17	<0.001*
Female	Age by MFH – CA	-0.712	2.55	0.011*

The correlation analysis summarized in Table 6 demonstrates a strong and statistically significant relationship between dental age estimated by the MFH method and chronological age across all gender groups. In male subjects (ρ = 0.974, n = 233, p < 0.001) and female subjects (ρ = 0.980, n = 155, p < 0.001), the method showed excellent reliability, with a slightly stronger correlation observed in females. When data from both sexes were combined, the correlation remained high (ρ = 0.979, n = 388, p < 0.001), underscoring the overall robustness of the MFH method in estimating chronological age.

**Table 5:** Correlation between chronological age and age estimated by MFH methods across gender groups. * p-value is statistically significant for male and female subjects both individually and combined and was calculated using Mann-Whitney to compare DA and CA. MFH: Moorrees, Fanning, and Hunt; DA: dental age; CA: chronological age.

Gender	Parameter	Value
Male	Rho value (ρ)	0.974
	p-value	<0.001*
	N	233
Female	Rho value (ρ)	0.980
	p-value	<0.001*
	N	155
Male and female	Rho value (ρ)	0.979
	p-value	<0.001*
	N	388

Linear regression analysis evaluating the relationship between dental age and chronological age is summarized in Table 7. The overall model (H1) revealed a strong positive association, with an intercept (a) of 0.546 and a slope (b) of 1.027, both statistically significant (p < 0.001).

**Table 6:** Linear regression for dental age and chronological age. p-value is statistically significant using Spearman's correlation comparing DA and CA; H1 refers to the regression model evaluating the relationship between dental age and chronological age. DA: dental age; CA: chronological age.

Model H1		
Intercept (a)	Slope (b)	p-value
0.546	1.027	<0.001

The regression equation, expressed as 𝑦 = 𝑎 + 𝑏𝑥, indicates that as dental age (x) increases, chronological age (y) increases proportionally (Figure 7). This model effectively quantifies the predictive relationship between dental development and actual age, reinforcing the utility of dental age as a reliable indicator of chronological age.

**Figure 1:** Linear regression for dental age and chronological age. This image has been created by the author, Shubham Srivastav.

When analyzed by gender, both male and female subjects exhibited similar linear relationships between dental age and chronological age. For male subjects, the linear regression yielded an intercept of 0.561 and a slope of 1.026 (Figure 8), while female subjects showed an intercept of 0.532 and a slope of 1.029 (Figure 9).

**Figure 2:** Linear regression for male dental and chronological age. This image has been created by the author, Shubham Srivastav.

**Figure 3:** Linear regression for female dental and chronological age. This image has been created by the author, Shubham Srivastav.

Both regressions were statistically significant (p < 0.001). As shown in Table 8, the slope values slightly greater than 1 indicate that dental age increases marginally faster than chronological age, though the relationship remains nearly linear in both groups.

**Table 7:** Linear regression for dental age and chronological age of male and female subjects. * p-value is statistically significant for male and female subjects using Spearman's correlation; H1 refers to the regression model evaluating the relationship between dental age and chronological age.

Model H1			
Gender	Intercept (a)	Slope (b)	p-value
Male	0.561	1.026	<0.001*
Female	0.532	1.029	<0.001*

Spearman’s rank correlation coefficients further confirmed a strong relationship between dental and chronological age: ρ = 0.974 for male subjects and ρ = 0.980 for female subjects (p < 0.001 for both). The slightly higher coefficient in females suggests a marginally stronger correlation in this group. These findings are consistent with the linear regression results and indicate a robust association between dental and chronological age across genders.

## Discussion

The present study evaluated the accuracy of the Moorrees, Fanning, and Hunt (MFH) method for estimating dental age (DA) and compared it with chronological age (CA) in a pediatric population. Age estimation is fundamental in pediatric dentistry, orthodontics, anthropology, and forensic investigations, especially when birth documentation is absent or unreliable. Dental development is considered a biologically stable marker, less influenced by environmental variables, making it a reliable tool for age estimation [14,15].

Our findings revealed a statistically significant underestimation of CA using the MFH method, with mean differences of -0.737 ± 2.17 years in male subjects and -0.712 ± 2.55 years in female subjects. The method demonstrated strong reliability, as indicated by high correlation coefficients (ρ = 0.974 for male subjects and ρ = 0.980 for female subjects). These findings are in agreement with those of Chatra et al., who reported an average underestimation of 3.0 years in male subjects and 2.9 years in female subjects among Indian children, with a correlation of r = 0.924 [16].

Similarly, Kuhnen et al. validated the MFH method in a Brazilian population, reporting its overall reliability while identifying developmental differences in specific teeth, such as canines, between sexes [17]. Phillips and van Wyk Kotze also found consistent underestimation across three South African ethnic groups, with an average deviation of 0.91 years, and emphasized the importance of population-specific adaptations [18].

Comparable underestimation was reported by Martínez and Ortega-Pertuz in a Venezuelan cohort, where the MFH method showed the largest mean discrepancy (-2.63 ± 2.09 years) when compared with other age estimation techniques [19]. In Iran, Naseh et al. observed a strong correlation (r = 0.931) between DA and CA using MFH, though again with a tendency to underestimate [20]. Kelmendi documented high reliability (r > 0.90) in a Kosovar population, further supporting our results [21].

According to Skanchy et al., neither the Demirjian method nor the Moorrees method provided accurate estimates of chronological age in their study of contemporary American Caucasian children aged nine to 14 years [22]. Conversely, AlOtaibi et al. found that among the various methods evaluated, Demirjian’s method was the most accurate for Saudi subjects, followed by the MFH methods [8]. In contrast, the methods developed by Nicodemo et al. and Chaillet et al. were identified as the least accurate [23,24].

Contrarily, Corral et al., in a Colombian study noted a slight overestimation of CA using the MFH method, suggesting that ethnic and environmental factors may influence the accuracy of this approach [25].

In the present study, regression analysis yielded slope values slightly greater than one (b ≈ 1.027), indicating that dental development advanced marginally faster than chronological progression. This pattern supports the consistent tracking of developmental maturity by the MFH method, though systematic underestimation necessitates calibration for specific populations.

The study encountered several significant limitations that influenced the accuracy and efficiency of dental age estimation. One of the primary challenges was the difficulty in precisely measuring the root lengths of maxillary and mandibular incisors, largely due to the absence of well-defined anatomical landmarks. This issue was particularly evident when comparing these teeth to mandibular molars and premolars, which typically offer clearer reference points for measurement. As a result, the evaluation of root development in these anterior teeth was less reliable. Additionally, in order to streamline the assessment process and avoid unnecessary delays, teeth with fully formed roots were excluded from the analysis. Since these teeth had completed their development, they were not expected to contribute meaningful information for age estimation. However, this exclusion may have limited the comprehensiveness of the assessment, as fully developed teeth could still offer contextual insights into overall dental maturation when interpreted alongside developing teeth [7].

While the MFH method demonstrates excellent reliability and correlation with CA, the observed consistent underestimation reinforces the need for regionally adjusted reference data or correction factors when applied in clinical or forensic contexts. Population-specific calibration may enhance its precision and utility in medico-legal applications.

## Conclusions

Based on the findings, the Moorrees, Fanning, and Hunt (MFH) method consistently underestimated dental age compared to chronological age in the Gandhinagar population, indicating notable limitations in its accuracy for this demographic. This systematic underestimation suggests that the MFH method, developed using data from a different population, may not adequately account for regional variations in genetic background, nutrition, health status, and socioeconomic factors that influence dental maturation. As a result, the applicability of this method in forensic and clinical settings within this population is constrained, highlighting the need for modified standards or alternative methods that offer greater precision in age estimation tailored to specific population characteristics.
